# Interpatient ECG Heartbeat Classification with an Adversarial Convolutional Neural Network

**DOI:** 10.1155/2021/9946596

**Published:** 2021-05-29

**Authors:** Jing Zhang, Aiping Liu, Deng Liang, Xun Chen, Min Gao

**Affiliations:** ^1^Department of Electrocardiogram, The First Affiliated Hospital of USTC, Division of Life Sciences and Medicine, University of Science and Technology of China, Hefei, Anhui 230001, China; ^2^School of Information Science and Technology, University of Science and Technology of China, Hefei 230027, China

## Abstract

Discovering shared, invariant feature representations across subjects in electrocardiogram (ECG) classification tasks is crucial for improving the generalization of models to unknown patients. Although deep neural networks have recently been emerging in extracting generalizable ECG features, they usually rely on labeled samples from a large number of subjects to guarantee generalization. Extracting invariant representations to intersubject variabilities from a small number of subjects is still a challenge today due to individual physical differences. To address this problem, we propose an adversarial deep neural network framework for interpatient heartbeat classification by integrating adversarial learning into a convolutional neural network to learn subject-invariant, class-discriminative features. The proposed method was evaluated on the MIT-BIH arrhythmia database which is a publicly available ECG dataset collected from 47 patients. Compared with the state-of-the-art methods, the proposed method achieves the highest performance for detecting supraventricular ectopic beats (SVEBs), which are very challenging to identify, and also gains comparable performance on the detection of ventricular ectopic beats (VEBs). The sensitivities of SVEBs and VEBs are 78.8% and 92.5%, respectively. The precisions of SVEBs and VEBs are 90.8% and 94.3%, respectively. With high performance in the detection of pathological classes (i.e., SVEBs and VEBs), this work provides a promising method for ECG classification tasks when the number of patients is limited.

## 1. Introduction

Classifying electrocardiogram (ECG) heartbeat is essential for cardiac diseases (e.g., cardiac arrhythmia) diagnosis. However, it is time consuming for cardiologists to inspect a long-term electrocardiogram (ECG) manually, making automatic ECG analysis useful. Currently, a large number of methods have been proposed for ECG classification. Two paradigms, known as intrapatient and interpatient paradigms, are usually adopted for evaluating ECG classification methods. In the intrapatient paradigm, the heartbeats from different patients are divided into the training and evaluation sets randomly. This evaluation paradigm is not highly reliable in the real world since the heartbeats from the same patients may be used for both the training and the testing, making the evaluation of the generalization of the classifier biased. In practice, an automatic ECG classification system should provide an accurate diagnosis for any unknown patient (patient not in the training set). The interpatient paradigm specifies that the heartbeats used for the training and the testing are from different individuals to obtain a more realistic evaluation. However, automatic interpatient ECG classification is a challenge today due to variations in ECG morphology and rhythm caused by individual physiological differences.

As illustrated in Figure 1, an ECG heartbeat mainly consists of a P wave, QRS complex wave, and *T* wave, which reflect electrical activities of depolarization and repolarization processes of the atria and ventricle. In general, a complete ECG classification system consists of three procedures: (1) ECG signal preprocessing, such as baseline wander removal and heartbeat segmentation; (2) feature extraction, mainly including morphological features [1–4], statistical features [5–7], P-QRS-T features [8–10], and wavelet features [11–13]; and (3) classification, such as support vector machine (SVM) [3, 9, 14, 15] and artificial neural network (ANN) [8, 16]. Chen et al. [9] combined projected ECG features and weighted RR interval features and then input these features into SVM for heartbeat classification. While their method yielded a high classification performance under the intrapatient evaluation paradigm, the sensitivity and precision metrics for detecting supraventricular ectopic beats were only 29.5% and 38.4% under the interpatient evaluation paradigm on the MIT-BIH arrhythmia database. Raj et al. [17] introduced a sparse representation technique to extract features representing ECG signals and used machine learning techniques (such as SVM and k-nearest neighbor) to classify these features, which obtain a good result in detecting supraventricular ectopic beats. Mondejar et al. [4] extracted morphological features and the features based on wavelets, high-order statistics, local binary patterns, and RR intervals. They proposed to feed each type of feature into a single SVM to train and obtain specific SVM models. Then, the predictions of these SVM models were combined to obtain the final prediction, which achieved an overall good performance for interpatient heartbeat classification. These methods rely on expert knowledge and experience for feature engineering. Thus, the classification performance could be very sensitive to the quality of extracted features.

Recently, many studies on ECG classification are increasingly focusing on deep learning due to its powerful ability for automatic feature learning and classification. When the training dataset is sufficient, deep neural networks (e.g., convolutional neural network (CNN)) are shown to be very predominant in classification tasks [18–22]. Hannun et al. presented a 34-layer deep CNN trained on 91232 ECG recordings collected from 53549 individuals, which achieved cardiologist-level accuracy in arrhythmia classification. However, complex models such as the CNN are prone to overfitting when the number of patients is limited (e.g., 47 different patients included in the MIT-BIH arrhythmia database), making it difficult for classifying the heartbeats of unknown patients. In fact, some deep learning-based methods [23–25] have achieved satisfactory results on small databases such as the MIT-BIH arrhythmia database for interpatient ECG classification. Li et al. [23] developed a multiscale convolutional neural network in which 3D features containing morphological characteristic, beat-to-beat correlation feature, and RR interval were taken as inputs. Niu et al. [24] proposed a deep-learning framework that introduces a symbolization approach to represent the rhythm and morphology of the heartbeat and feeds the symbolic representation into a multiperspective convolutional neural network. However, current methods lacked explicit mechanisms to explore ECG feature invariance across subjects. They usually stand on the assumption that their proposed models can intrinsically learn generalizable features during training. This implicit learning is naturally restrained by the amount of individual ECG data. Therefore, how to explicitly learn invariant representations against intersubject variations is a critical issue, especially when the number of patients is limited.

In this paper, we propose an adversarial ECG heartbeat classification framework based on a convolutional neural network, as illustrated in Figure 2. The framework integrates adversarial learning into a convolutional neural network, which extends deep-learning models for ECG identification tasks. The adversarial CNN is composed of an encoder, classifier, and adversary networks. The encoder network extracts features from ECG heartbeat signals and corresponding RR intervals. The classifier and adversary networks are responsible for maximizing the class labels prediction and minimizing the subject ID identification. By this adversary game, the encoder is trained to learn subject-invariant, class-discriminative features. The proposed method was evaluated on the MIT-BIH arrhythmia database which is a publicly available ECG dataset collected from 47 patients. Ablation studies show that our adversarial subject-invariant feature learning significantly enhances interpatient ECG heartbeat classification accuracy compared to conventional deep-learning methods.

The main contributions of this paper are concluded as follows:

1. Our goal is that the features learned by a deep-learning model can generalize to unknown patients well for ECG identification/classification tasks. To this end, a deep-learning-based ECG heartbeat classification framework is proposed for tackling the learning of generalizable features. Specifically, we introduce an adversary loss into the convolutional neural network, encouraging the model to learn subject-invariant, class-discriminative representations from an insufficient number of subjects through the adversary game.
2. The experiments on the publicly available and commonly used dataset, MIT-BIH database, demonstrate that the proposed method can achieve the state-of-the-art performance on the detection of pathological classes when the number of subjects is limited.

## 2. Method

### 2.1. Problem Description

Let {(**X**_*i*_, *y*_*i*_, *s*_*i*_)}_*i*=1_^*n*^ indicate the training set, with **X**_*i*_ denoting the original ECG heartbeat, *y*_*i*_ ∈ {0,1,…, *C* − 1} denoting the class label of **X**_*i*_, and *s*_*i*_ ∈ {1,…, *S*} denoting the subject identification (ID) number of **X**_*i*_. The reasonable assumption here is ECG data **X** being jointly dependent on class labels *y* and subject IDs *s*. The task of ECG classification is to predict *y* given **X**. In the real world, this task requires the predictions invariant to *s*, namely, a generalizable model across subjects is necessary. In this study, we regard *s* as the nuisance variable and aim to develop a convolutional neural network model to learn generalizable features across subjects that are invariant to *s*.

### 2.2. Data Preprocessing and Feature Extraction

All original ECG recordings are preprocessed to generate the input of the proposed adversarial convolutional neural network, as presented in Figure 2(a). First, we segment the original ECG recordings into heartbeats according to the locations of *R* peaks annotated by the MIT-BIH arrhythmia database. Specifically, the 50 points after the previous *R* peak and the 100 points after the current *R* peak are taken as a heartbeat. This segmentation allows heartbeats to contain a more robust P-QRS-T complex waveform since the heart rate is constantly changing, and the fixed starting point relative to the current *R* peak may introduce disturbance information (heartbeats with a short RR interval) or lose information (heartbeats with a wide waveform). Our segmentation will result in heartbeats of different lengths; however, CNNs fail to accept the varied-length input. Therefore, in the second step, we resample all heartbeats to the same length 128. Third, the average of all heartbeat segments is subtracted to suppress the baseline wander.

In addition to the preprocessed heartbeat signal, the heartbeat rhythm (RR interval information) is extracted as another part of the input, as shown in Figure 2(b). The pre-RR interval (the interval between the current *R* peak and the previous one) is a typical RR interval feature, which generally can distinguish arrhythmias from normal heartbeats of a person [27]. However, the pre-RR interval distribution of arrhythmic heartbeats may overlap with that of normal heartbeats as the individual basic heart rate is different, especially for the patient population. To eliminate the overlap, we extract the pre-RR ratio (the ratio of the current pre-RR interval to the average of all pre-RR intervals of the corresponding recording) to unify everyone's basic heart rate. Furthermore, the near-pre-RR ratio (the ratio of the current pre-RR interval to the average of the previous ten pre-RR intervals) is also extracted since the individual basic heart rate changes with mood and movement state [1]. To build the input of the adversarial convolutional neural network, we duplicate these two scalar features as vectors with a length of 128 and then concatenate with the preprocessed heartbeat signal.

### 2.3. Adversarial Model Learning

The proposed adversarial ECG heartbeat classification model mainly consists of three parts: an encoder, classifier, and adversary subnetworks, as illustrated in Figure 2(c). The encoder network $f\left(\tilde{X};\theta_{e}\right)$ parameterized by *θ*_*e*_ is used to learn representations *h*. In implementation, the convolution neural network is as the encoder, which is detailed in Section 2.4. The encoder outputs the representations *h*, and *h* are fed into the classifier *q*_*θ*_*c*__(*y|h*) parameterized by *θ*_*c*_ and the adversary network *q*_*θ*_*a*__(*s|h*) parameterized by *θ*_*a*_ separately. The classifier and adversary, consisting of a fully connected layer with softmax function, are used to classify the representations *h* into heartbeat classes *y* and subject IDs *s*, respectively. To eliminate interferences caused by *s* that are embedded in *h*, we present an adversarial game. Here, the adversary is trained to predict subject IDs *s* by maximizing the likelihood *q*_*θ*_*a*__(*s|h*), while at the same time, the encoder is trained to conceal information regarding *s* within *h* by minimizing this likelihood and retain sufficient discriminative information for the classifier to estimate class labels *y* by maximizing *q*_*θ*_*c*__(*y|h*). Overall, we train the encoder, classifier, and adversary networks jointly towards the objective:

(1) $$\begin{array}{c} {\hat{\theta }}_{e},{\hat{\theta }}_{c},{\hat{\theta }}_{a}=\arg\underset{\theta_{e},\theta_{c}}{\min}\underset{\theta_{a}}{\max}L\left(\theta_{e},\theta_{c},\theta_{a}\right), \end{array}$$

where *L* is the cross-entropy loss function, defined by

(2) $$\begin{array}{c} L=E_{h}E_{y}\left[-\log\;q_{\theta_{c}}\left(y|h\right)\right]+\lambda E_{h}E_{s}\left[\log\;q_{\theta_{a}}\left(s|h\right)\right], \end{array}$$

where *λ* denotes the adversarial weight trading off between stronger invariance with task-discriminative performance. A higher *λ*(>, 0) enhances invariance to subjects, whereas *λ* < 0 forces the encoder to learn features that are discriminative for class labels, as well as subject IDs, which is not expected in our ECG classification task.

### 2.4. Convolutional Network Architecture

The ECG feature encoder is composed of 7 convolution layers and three spatiotemporal attention modules in total. The specific configuration of the encoder network is shown in Table 1. Following the first convolution layer, three residual convolution blocks with average pooling shortcuts are built to facilitate the optimization of the network and gain classification accuracy. The second (the last) convolution layer of each residual block uses the dilation rate of 3 to enlarge the receptive field without increasing the parameter amount. After all convolution layers, batch normalization (BN) [28] is used to accelerate model convergence by renormalizing the distribution of training minibatch. The Rectified Linear Unit (ReLU) function [29] is applied to activate the output of each BN layer, which could prevent the vanishing gradient problem well. Furthermore, we introduce a spatiotemporal attention mechanism [30], including spatial and temporal attention modules, which is embedded after each residual convolution block. This mechanism could focus on more informative features by assigning different weights to both channels and temporal segments of the feature map.

Learned representations *h* by the encoder network are input to the classifier and adversary for task discrimination (heartbeat class) and subject ID discrimination. Both the classifier and adversary consist of a fully connected layer with *C* and *S* softmax units, respectively, to output normalized log-probabilities that will be used to calculate the loss *L* in equation (2).

## 3. Experimental Studies and Results

### 3.1. Dataset

The MIT-BIH arrhythmia database [31] is used for evaluating the performance of the proposed method. This database consists of 48 two-lead ambulatory ECG recordings collected from 47 individuals, where recordings 201 and 202 were obtained from the same subjects. Each recording lasts about 30 minutes and is sampled at 360 Hz. According to ANSI/AAMI EC57:1998 [32], all heartbeats can be grouped into five superclasses: heartbeats originating in the sinus node (N), supraventricular ectopic beats (SVEBs or S), ventricular ectopic beats (VEBs or V), fusion beats (F), and unknown beat type (*Q*).

Following the AAMI-recommended practice, four paced recordings are not used. To obtain a more realistic evaluation, De Chazal et al. [33] recommended dividing the remaining 44 recordings into DS1 and DS2 sets for the training and test, respectively. This division splits the recordings by considering the identification of patients and the balance of classes, which guarantees that the heartbeats in the training and testing sets are from different patients. The detailed heartbeat distribution used in this paper is shown in Table 2.

### 3.2. Training Setting

20% of the training data is randomly chosen as the validation data, and the remaining data are used as the training samples. We set the adversarial weight *λ* to 0.005 by finetuning this parameter. The proposed adversarial deep-learning framework is trained by using an adaptive moment estimation (Adam) optimizer [34] with an initial learning rate of 0.001. During training, the model parameters are updated iteratively based on batches of 128 training samples. When the loss *L*_*c*_ of the validation data remains undeclined for 10 epochs, the learning rate decreases to 0.0001, while for 20 epochs, the training will terminate. The best-performing model on validation data for heartbeat classification is saved.

### 3.3. Evaluation Metrics

Four typical metrics, including accuracy (Acc), sensitivity (Sen), precision (Pre), and *F*_1_ score, are used to measure the classification performance of the proposed method. Here, accuracy measures the overall classification performance of the proposed method, whereas sensitivity and precision metrics are calculated for each specific class. *F*_1_ score is the harmonic mean of precision and recall. These metrics are defined as

(3) $$\begin{array}{c} \text{Acc}=\frac{\text{TP}+\text{TN}}{\text{TP}+\text{TN}+\text{FP}+\text{FN}},\\ \text{Sen}=\frac{\text{TP}}{\text{TP}+\text{FN}},\\ \text{Pre}=\frac{\text{TP}}{\text{TP}+\text{FP}},\\ F_{1}=\frac{2\times \left(\text{Precision}\times \text{Recall}\right)}{\text{Precision}+\text{Recall}}, \end{array}$$

where TP, TN, FP, and FN refer to the sample number of true positive, true negative, false positive, and false negative, respectively. Actually, the accuracy metric is largely dominated by the class (class N) with larger number of samples. To saliently reflect the classification performance of a model for pathological classes S and V, in addition to class-level *F*_1_ scores *F*_1_*S*__ and *F*_1_*V*__ for these two classes, we further define the average *F*_1_ score of S and V as

(4) $$\begin{array}{c} \text{pat}\_F_{1}=\frac{F_{1_{S}}+F_{1_{V}}}{2}. \end{array}$$

### 3.4. Classification Performance

Following the AAMI recommendation, we particularly focus on the classification performance of classes S and V since the proportions of training samples for these two arrhythmic classes are much higher (2.8% and 7.0%) and cover the majority of arrhythmias. The training samples of classes F and *Q* are very scarce (0.8% of the whole dataset), and the detection accuracy is usually pretty low in the literature.  Figure 3 presents the confusion matrix for the heartbeat classification results on DS2, where the darker color indicates the more accurate prediction. Overall, the proposed method achieves high ECG heartbeat classification performance on classes N, S, and V. Most instances of classes N, S, and V are correctly classified. Nevertheless, the classification of classes F and *Q* is unsatisfactory. It is mainly due to the considerable small number of training samples for these two classes, as seen in Table 2. Furthermore, we evaluate the record-level classification results of the proposed method on DS2, as shown in Table 3. 18 out of 22 recordings attain an accuracy of above 90%. The classification accuracies of other 4 recordings 105, 202, 213, and 214 are 87.9%, 85.4%, 88.7%, and 65.2%, respectively. The overall classification performance of class V (92.5% sensitivity and 94.3% precision) is better than that of class S (78.8% sensitivity and 90.8% precision). This is partially because class S has a smaller sample size but more subclasses than class V.

### 3.5. Performance Comparison

Table 4 compares the interpatient heartbeat classification performance of several other methods and ours. Same as our evaluation scheme, these methods trained their models using the DS1 set and were evaluated on DS2, ensuring a fair comparison. As mentioned above, we focus more on the classification performance for classes S and V rather than the overall accuracy which is mainly governed by class N with the very large instances (90% of the whole dataset). In clinic, missing diagnosis is particularly serious, which can be reflected by sensitivity metric. Also, precise diagnosis is necessary. Thus, the comparison focuses on *F*_1_ scores for pathological classes S and V, taking into account both sensitivity and precision metrics. Moreover, it is easy to make a comparison of a single metric between different methods. Thus, *pat*_*F*_1_ score, which is the average value of *F*_1_*S*__ and *F*_1_*V*__ for pathological classes S and V, is used as the final metric.

In [3, 4, 17, 35], the traditional ECG classification pipeline is adopted, which extracts features based on experiences from raw or preprocessed ECG signals and then inputs these extracted features into a classifier. Compared with these methods, the proposed method has a higher pat_*F*_1_ score of 11.4%–25%. [23, 24], and ours utilized a deep-learning model to automatically extract useful features and classification, coupled with some hand-craft features. The proposed adversarial CNN outperforms [23, 24] by 17.2% and 5.8% pat_*F*_1_ scores, respectively. It can be observed that the proposed method achieves the highest pat_*F*_1_ score. On the whole, the proposed method has an advantage in detecting pathological classes, especially class S which is challenging to identify in the MIT-BIH dataset, and also obtains a satisfactory performance (*F*_1_ score of >90%) in detecting class V.

## 4. Discussion

### 4.1. Effects of RR Ratio Features

To explore the effect of the pre-RR ratio and near-pre-RR ratio for classifying arrhythmias (i.e., classes N, S, V, F, and Q), the box plots that show the distribution of these two RR ratios among classes are given as Figure 4. It is obviously observed that two RR ratios can distinguish pathological classes S and V from class N well. Nevertheless, it is difficult to distinguish between S and V. This is reasonable due to some shared characteristics between pathological ECG recordings, such as too fast or too slow rhythm. Therefore, additional ECG feature learning by other techniques is necessary, such as deep learning used in this paper. Class F, which is the fusion of ventricular and normal beats, has a distribution of two RR ratios close to that of class N. Class *Q* consists of unknown beats. Thus, its RR ratios span a wide range of distribution. The comparison for classification performance between with/without the pre-RR ratio and near-pre-RR ratio is shown in Table 5. The experimental results demonstrate that these two RR ratio features greatly improve the sensitivity and precision in detecting pathological classes S and V by providing more prior knowledge about heart rhythms to the deep network.

### 4.2. Regular CNN vs. Adversarial CNN

Here, the regular CNN indicates the encoder-classifier network. We remove the adversary subnetwork from the proposed framework to validate the effectiveness of adversarial learning. The same data processing, feature extraction, and experiment setting are performed between the regular CNN and the proposed adversarial CNN. The comparison for classification performance is shown in Table 6. It is obvious that the proposed adversarial CNN is far superior to the regular CNN, except that the precision metric for class V is slightly lower. The regular CNN is data driven in essence. However, the ECG recordings provided in the MIT-BIH database are collected from an insufficient number of subjects. Therefore, it is challenging to capture the robust features against intersubject variabilities using the regular CNN, and the learned features could be subject related. On the contrary, the proposed adversarial CNN works out concealing the information of subject IDs by the adversarial game. The experimental result suggests that the adversarial learning can significantly facilitate learning generalizable features across subjects that are invariant to subjects.

### 4.3. Choosing the Adversarial Weight Parameter

The adversarial weight *λ* makes a tradeoff between the invariance to subjects and task-discriminative performance. A very strong *λ* will promote the encoder to learn subject-invariant information. However, increasing *λ* can result in losing task-discriminative information. Here, we implemented several experiments to analyze the effect of different adversarial weights *λ*.  Table 7 shows experimental results. For class N, the sensitivity and precision of different *λ* are all higher than 90%, which should be attributed to a large sample number of class N. For classes S and V, it can be seen that the performance of a higher *λ* is low (when *λ*=0.01, 0.05, and 0.1). When *λ*=0.005, the overall performance is the highest.

### 4.4. Visualization of Learned Features

The t-distributed stochastic neighbor embedding (t-SNE) [36] can reduce high-dimensional data to a two-dimensional map nonlinearly. Here, we applied t-SNE to evaluate the proposed method visually. The preprocessed heartbeat segment is 256-dimensional vectors (the length is 128 and the channel number is 2). Combining RR ratio features with the heartbeat segment, 768-dimensional vectors (two RR ratio features and the heartbeat segment are all 256-dimensional vectors) were used as the input of the proposed adversarial CNN. We extracted the outputs from different layers. The visualizations are shown in Figure 5. The sample size of class N was reduced in the figures for a good visualization. It can be observed from Figures 5(a) and 5(b) that no obvious clusters exist in the input feature vectors. As the layer deepens, the clusters become apparent (Figures 5(c) and 5(f)). However, in the first three residual blocks, the clustering of each class is still separated. This means that these feature vectors fail to distinguish classes N, S, V, F, and *Q* well and further nonlinear operations are required. For the feature vectors output by the global average-pooling layer (Figure 5(f)), the clustering is very apparent. Figure 5(f) demonstrates that the extracted features by the proposed method are discriminative to classify multiclass arrhythmias. It is noted that each class may contain multiple clusters. This is because each class consists of multiple subclasses in which some features are different. For example, bundle branch block beat and normal beat belong to class N, while they have different QRS complex durations.

## 5. Conclusions

This paper presents a CNN-based adversarial deep-learning framework for interpatient heartbeat classification using a small subject number of ECG signals. The proposed framework consists of an encoder, classifier, and adversary networks. The encoder is used to learn representations from input data generated by raw signal preprocessing and feature extraction procedures. Then, these representations are fed separately into the classifier and adversary to classify heartbeats and subject IDs. The overall framework is trained by minimizing the heartbeat classification loss and maximizing the subject ID identification loss, enforcing the encoder to conceal information regarding subject IDs and retain sufficient discriminative information for task (heartbeat) classification. The proposed framework can help to eliminate the interpatient variability and obtain invariant representations across subjects by utilizing the adversarial learning. Therefore, it is especially suitable for ECG classification tasks with an insufficient number of patients.

## Figures and Tables

**Figure 1:** A typical ECG heartbeat waveform [26].

**Figure 2:** The overall framework for interpatient heartbeat classification. (a) Data preprocessing including heartbeat segmentation operation is performed given an original ECG signal. (b) The feature extraction process. (c) The adversarial convolutional neural network, consisting of an encoder, classifier, and adversary subnetworks. The adversarial CNN is jointly trained towards the objective defined by equation (1).

**Figure 3:** Confusion matrix of the proposed method.

**Figure 4:** (a) The box plot of the pre-RR ratio for different classes. (b) The box plot of the near-pre-RR ratio for different classes.

**Figure 5:** The t-SNE visualization for input feature vectors and middle-layer outputs for the DS2 test set. (a) 256 D heartbeat segment, (b) 768-D input feature vectors, (c) outputs from the 1st block, (d) outputs from the 2nd block, (e) outputs from the 3rd block, and (f) the final feature vectors.

**Table 1:** The configuration for the encoder network.

Layer	Output size	Kernel size	Padding	Strides	Dilation rate
Inputs	(3 × 128 × 2)	—	—	—	—
Conv layer1	(1 × **1**26 × 16)	(3 × 3)	Valid	1	1
Residual block1 layer1	(1 × 126 × 16)	(1 × 3)	Same	1	1
Residual block1 layer2	(1 × 126 × 16)	(1 × 3)	Same	1	3
Spatioattention module	(1 × 126 × 16)	—	—	—	—
Residual block2 layer1	(1 × 63 × 64)	(1 × 3)	Same	2	1
Residual block2 layer2	(1 × 63 × 64)	(1 × 3)	Same	1	3
Spatioattention module	(1 × 63 × 64)	—	—	—	—
Residual block3 layer1	(1 × 32 × 64)	(1 × 3)	Same	2	1
Residual block3 layer2	(1 × 32 × 64)	(1 × 3)	Same	1	3
Global average pooling	(64)	—	—	—	—

**Table 2:** Distribution of the heartbeats in DS1 and DS2.

AAMI	MIT-BIH heartbeat classes	#DS1	#DS2	#DS1 + DS2
**N**		45683	44082	89765
	Normal beat (N)	37951	36304	74255
	Left bundle branch block beat (L)	3940	4109	8049
	Right bundle branch block beat (R)	3760	3456	7216
	Atrial escape beat (e)	16	0	16
	Nodal (junctional) escape beat (j)	16	213	229

**S**		944	1831	2775
	Atrial premature beat (A)	810	1730	2540
	Aberrated atrial premature (a)	100	50	150
	Nodal (junctional) premature beat (J)	32	51	83
	Supraventricular premature beat (S)	2	0	2

**V**		3778	413	8
	Premature ventricular contraction (V)	3673	3207	6880
	Ventricular escape beat (E)	105	1	106

**F**	Fusion of ventricular and normal beat (F)	413	388	801
**Q**	Unclassified beat (Q)	8	7	15
**Total**		**5082**	**49516**	**100332**

**Table 3:** Record-level performance of the proposed method on DS2.

	Number of heartbeats				N		S		V		Overall
Recording	All	N	S	V	Sen	Pre	Sen	Pre	Sen	Pre	Acc
100	2264	2231	32	1	100.0%	99.3%	53.1%	100.0%	100.0%	100.0%	99.3
103	2075	2073	2	0	99.7%	99.9%	0.0%	0.0%	—	—	99.6
105	2563	2517	0	41	88.6%	99.1%	—	—	56.1%	42.6%	87.9
111	2115	2114	0	1	100.0%	100.0%	—	—	100.0%	100.0%	100.0
113	1786	1780	6	0	100.0%	99.7%	0.0%	0.0%	—	—	99.7
117	1526	1525	1	0	100.0%	100.0%	100.0%	100.0%	—	—	100.0
121	1854	1852	1	1	99.8%	99.9%	0.0%	0.0%	100.0%	25.0%	99.8
123	1509	1506	0	3	95.5%	100.0%	—	—	100.0%	100.0%	95.5
200	2592	1739	30	821	99.4%	95.1%	0.0%	0.0%	92.0%	98.7and	95.8
202	2127	2052	55	19	86.9%	98.3%	27.3%	100.0%	94.7%	66.7%	85.4
210	2561	2415	22	194	96.0%	97.4%	27.3%	28.6%	74.2%	100.0%	93.4
212	2739	2739	0	0	100.0%	100.0%	—	—	—	—	100.0
213	3242	2632	28	220	99.8%	89.2%	0.0%	0.0%	77.3%	94.4%	88.7
214	2253	1995	0	255	61.0%	99.7%	—	—	99.2%	98.8%	65.2
219	2145	2073	7	64	99.1%	99.4%	0.0%	0.0%	92.2%	77.6%	98.6
221	2418	2024	0	394	100.0%	99.8%	—	—	98.7%	100.0%	99.8
222	2474	2265	209	0	98.2%	94.7%	40.7%	68.5%	—	—	93.3
228	2044	1679	3	362	95.1%	98.3%	0.0%	0.0%	92.5%	81.5%	94.5
231	1563	1560	1	2	100.0%	99.9%	0.0%	0.0%	50.0%	100.0%	99.9
232	1772	395	1377	0	99.0%	87.7%	95.6%	99.8%	—	—	96.4
233	3070	2225	7	827	99.7%	98.9%	28.6%	100.0%	98.1%	98.7%	98.8
234	2744	2691	50	3	100.0%	98.2%	0.0%	0.0%	100.0%	100.0%	98.2
Total	49516	44082	1831	3208	96.2%	98.0%	78.8%	90.8%	92.5%	94.3%	94.7

**Table 4:** Performance comparison between the previous works with ours on DS2.

Work	Year	Method	*F*_1_*S*__	*F*_1_*V*__	pat_*F*_1_
[3]	2017	Features: temporal vector cardiogram + complex network	57.1%	70.7%	63.9%
		Classifier: SVM			

[17]	2018	Features: features by sparse decomposition	60.8%	83.8%	72.3%
		Classifier: least-square twin SVM			

[23]	2019	Multiscale CNN + RR features + beat-to-beat correlation	50.7%	92.6%	71.7%
[4]	2019	Features: wavelets + local binary patterns + higher-order statistics	60.7%	**94.3%**	77.5%
		+amplitude values			
		Classifier: SVMs			

[24]	2020	Multiperspective CNN + symbol representations + RR features	76.5%	89.7%	83.1%
[35]	2021	Features: signal morphology + higher-order statistics	52.2%	90.8%	71.5%
		+RR features			
		Classifier: linear discriminant			

Proposed		Adversarial CNN + RR features	**84.4%**	93.4%	**88.9%**

pat_*F*_1_ score is the average value of *F*_1_*S*__ and *F*_1_*V*__ for pathological classes S and V, defined as equation (4).

**Table 5:** Performance comparison between with/without RR ratio features on DS2.

Features	Acc	Sen_*N*_	Pre_*N*_	Sen_*S*_	Pre_*S*_	Sen_*V*_	Pre_*V*_
Without RR ratios	94.0	**98.7%**	95.0%	6.3%	42.2%	88.7%	91.3%
With RR ratios	**94.7**	96.2%	**98.0%**	**78.8%**	**90.8%**	**92.5%**	**94.3%**

**Table 6:** Performance comparison between the regular CNN with the proposed adversarial CNN on DS2.

Framework	Acc	Sen_*N*_	Pre_*N*_	Sen_*S*_	Pre_*S*_	Sen_*V*_	Pre_*V*_
Regular CNN	93.9	95.9%	97.6%	69.1%	82.1%	89.9%	85.7%
Adversarial CNN	**94.7**	**96.2%**	**98.0%**	**78.8%**	**90.8%**	**92.5%**	**94.3%**

**Table 7:** Performance comparison for different adversarial weights on DS2.

Parameter setting	Acc (%)	Sen_*N*_	Pre_*N*_	Sen_*S*_	Pre_*S*_	Sen_*V*_	Pre_*V*_
*λ*=0.001	93.9	95.9%	97.6%	69.1%	82.1%	89.9%	85.7%
*λ*=0.005	94.7	96.2%	**98.0%**	**78.8%**	**90.8%**	**92.5%**	**94.3%**
*λ*=0.01	**95.3**	**98.0%**	96.9%	60.3%	81.6%	89.3%	90.3%
*λ*=0.05	91.5	93.4%	97.5%	60.7%	74.6%	92.5%	69.3%
*λ*=0.1	93.5	95.5%	97.4%	67.7%	81.7%	92.0%	70.6%

## Data Availability

The MIT-BIH Arrhythmia Database used to support the findings of this study is publicly available and can be downloaded at https://physionet.org/content/mitdb/1.0.0/.
